# LINC00035 Transcriptional Regulation of SLC16A3 via CEBPB Affects Glycolysis and Cell Apoptosis in Ovarian Cancer

**DOI:** 10.1155/2021/5802082

**Published:** 2021-10-11

**Authors:** Shuyan Yang, Jing Wang, Rongjie Cheng, Bo Pang, Pengcheng Sun

**Affiliations:** Department of Obstetrics and Gynecology, The Fourth Affiliated Hospital of Harbin Medical University, No. 37, Yiyuan Street, Nangang District, Harbin 150001, Heilongjiang, China

## Abstract

**Objective:**

Ovarian cancer (OC) represents the most lethal gynecologic malignancy globally. Over the decades, lncRNAs have been considered as study focuses due to their genome-wide expression through multiple mechanisms in which regulation of target gene transcription through interaction with transcription factors or epigenetic proteins is proven. In the present work, we focus on the functional role of LINC00035 in OC and its regulation mechanism on gene expression.

**Methods:**

We collected OC tissues and adjacent tumor-free tissues surgically resected from 67 OC patients. Cultured human OC cell lines SKOV3 and A2780 were assayed for their viability, migration, invasion, apoptosis *in vitro* using CCK-8 assays, transwell assays, and flow cytometric analysis. OC cell tumorigenesis *in vivo* was evaluated by mouse xenograft experiments. Glycolysis was evaluated by glucose uptake, lactate release, and ATP production assays. Luciferase activity assay, RNA immunoprecipitation (RIP), and RNA pull-down were performed to confirm the interactions among LINC00035, CEBPB, and SLC16A3.

**Results:**

LINC00035 was upregulated in OC tissues. LINC00035 knockdown was shown to repress SKOV3 and A2780 cell viability, migration, invasion, induce their apoptosis, and reduce glucose uptake, lactate release, and ATP production. LINC00035 could recruit CEBPB into the SLC16A3 promoter region, thus increasing the SLC16A3 transcription. SLC16A3 was upregulated in OC tissues. SLC16A3 knockdown exerted similar effects on SKOV3 and A2780 cells as LINC00035 knockdown. Rescue experiments found SLC16A3 overexpression resisting to LINC00035 knockdown on SKOV3 and A2780 cell viability, migration, invasion, apoptosis, glucose uptake, lactate release, and ATP production. Results also showed LINC00035 knockdown could inhibit OC cell tumorigenesis *in vivo*.

**Conclusion:**

The study reveals that LINC00035 promotes OC progression by regulating glycolysis and cell apoptosis through CEBPB-mediated transcriptional promotion of SLC16A3.

## 1. Introduction

Ovarian cancer (OC) is the third most common gynecologic malignancy and one of the leading causes of cancer death among women around the world [1]. OC is considered to be a heterogeneous malignant tumor with unique genomic characteristics. Histologically, it can be divided into five different subtypes at least [2]. The report of Global Cancer Statistics 2020 estimated that the incidence and mortality of OC accounts for 1.6% and 2.1%, respectively [3]. Due to less early clinical features and the presence of metastatic and invasive cancer cells in most patients at the time of diagnosis, OC remains one of the most challenging malignancies to manage [4]. Most women with serous carcinomas are diagnosed at stage III (51%) or IV (29%), with a high rate of relapse and metastasis into the abdominal cavity [5]. A large-scale study of OC screening has shown that only using ultrasound or CA125 test for screening every year and, if necessary, follow-up with ultrasound fails to decrease mortality in the general population. Despite more early diagnosis by screening, the increase was not sufficient to significantly improve survival [6, 7]. Given that various factors involving frequent recurrence, late stage during initial diagnosis, the presence of resistance to drugs, and adverse reaction to chemotherapeutic regimens occur in most of the patients, it has become imperative to extensively elucidate the underlying mechanisms behind OC development. Long noncoding RNAs (lncRNAs), a subgroup of RNAs (>200 nucleotides in length), engage in OC initiation, drug resistance, and progression [8, 9]. LINC00035, located on the human chromosome 7q11.23, with another known name ABHD11-AS1, has been widely confirmed as an oncogene, showing different power of gene control, including epigenetic, transcription, or posttranscriptional control in many types of human cancers, such as gastric cancer [10], pancreatic cancer [11], endometrial carcinoma [12], thyroid cancer [13], lung cancer [14], and breast cancer [15].

LncRNAs interact with a variety of transcription factors to modulate gene expression and then participate in cell growth and apoptosis [16]. The transcription factor CCAAT/enhancer-binding protein beta (CEBPB) is required for maintenance of the tumor-initiating capacity and invasion ability in several tumors, including hepatocellular carcinoma [17], glioblastoma [18], and breast cancer [19]. SLC16A3 is a member of the SLC16 gene family that has fourteen members among which SLC16A1, SLC16A3, SLC16A7, and SLC16A8 encode proton-coupled monocarboxylate transporters MCT1, MCT4, MCT2, and MCT3, respectively [20]. SLC16A3 has the ability to catalyze the proton-linked transport of monocarboxylates such as l-lactate, pyruvate, and ketone bodies across the plasma membrane, which was recognized as glycolysis-related gene signature in human cancers [21, 22]. The LncMAP database (http://bio-bigdata.hrbmu.edu.cn/LncMAP/) shows LINC00035 regulates transcription factor CEBPB and its downstream gene SLC16A3 in OC. Based on the aforementioned data, we therefore speculate whether there is a promising correlation among LINC00035, CEBPB, and SLC16A3 in OC.

## 2. Materials and Methods

### 2.1. Human Tissue Specimen

We collected OC tissues and adjacent tumor-free tissues surgically resected from 67 OC patients who were admitted into our hospital in the time duration from January 2020 to December 2020. No patients had received radiotherapy, chemotherapy, or immunotherapy before surgery. Signed informed consents were obtained from all participants. The study was approved by the Institutional Review Board of our hospital. Experiments involving human beings were performed in strict accordance with the Declaration of Helsinki.

### 2.2. Cell Culture and Transient Transfection

Under the conditions of humidity of 5% CO_2_ and temperature of 37°C, IOSE80 used as normal ovarian epithelial cells and Caov-3, A2780, SKOV3, and CoC1 used as human OC cell lines (ATCC, USA) were grown in the RPMI1640 with 15% fetal bovine serum (FBS) (Gibco, USA). To construct OC cells with LINC00035 overexpression and knockdown, CEBPB overexpression and knockdown, SLC16A3 overexpression and knockdown, siRNA targeting LINC00035, the expression vector containing the full-fragments of LINC00035, siRNA targeting CEBPB, the expression vector containing the full-fragments of CEBPB, siRNA targeting SLC16A3 and the expression vector containing the full-fragments of SLC16A3 were delivered into selected OC cells by mean of lipofectamine 2000 reagent transfection (Invitrogen, USA). Cell transfection was performed lasting for 24–48 h.

### 2.3. Quantitative Real-Time Polymerase Chain Reaction (qRT-PCR)

After total RNA extractions from tissue and cells by using Trizol reagents (Invitrogen), cDNA was generated according to the manuals of the PrimeScript RT reagent Kit (Takara, Japan). The SYBR®Premix ExTaqTM II (RR820A, Takara) kit and the ABI PRISM®7300 System (ABI, USA) were applied to complete the qRT-PCR. Data were relative to the expression of a reference gene GADPH and analyzed using the 2^−ΔΔCt^ method. The primers of LINC00035, SLC16A3, and GADPH were synthesized by RiboBio (Guangzhou, China). The primer sequences of LINC00035 were 5′-TCCAGACAAGACTTGGTCGC-3' (forward) and 5′-CAGCTGGTTGTGTGGCTTTC-3' (reverse), of SLC16A3 were 5′-CTTCCCGTCAGACGCCC-3' (forward) and 5′-GTGTTCAGTACCAGCCCTGT-3' (reverse), and of GADPH were 5′-ATGGAGAAGGCTGGGGCTC-3' (forward) and 5′-AAGTTGTCATGGATGACCTTG-3' (reverse).

### 2.4. CCK-8 Assays

A2780 and SKOV3 cells were incubated with 3 × 10^3^ cells per well in the 96-well plate. Upon incubation at different time points, 0, 1, 2, and 3 d, each well reacted with the addition of CCK-8 reaction solution (Dojindo, Kumamoto, Japan). Another 2h incubation continued. The optical value was obtained at 450 nm.

### 2.5. Transwell Migration and Invasion Assays

A2780 and SKOV3 cells (6 × 10^4^ cells for each) were suspended in 200 *μ*L serum-free medium and supplemented into the apical chamber of the transwell system (Corning-Costar, Cambridge, MA) uncoated (for migration) or coated (for invasion) with Matrigel (BD Biosciences, San Jose, CA). Additional 700 *μ*L DMEM with 10% FBS was added into the basolateral chamber. Following 24-hour incubation, A2780 and SKOV3 cells were transferred from the apical chamber into the basolateral one, followed by addition of methanol and 0.1% crystal violet. The number of migrating or invasive cells was photographed under an inverted microscope and also calculated flow cytometric analysis.

A2780 and SKOV3 cells were suspended in the DMEM to adjust the density into 1 × 10^6^ cells/mL. The cell suspensions reacted with the addition of 5 *μ*l Annexin V and 5 *μ*l propidium iodide (PI). Apoptotic A2780 and SKOV3 cells were analyzed using a flow cytometer (FACScan®) equipped with Cell Quest software (BD Biosciences).

### 2.6. Immunoblotting Analysis

After 10% SDS-PAGE separation, extracted total protein was wet-transferred to the PVDF membrane (Sigma-Aldrich, USA). Immunoblots were generated after addition of primary antibodies: anti-bcl-2 antibody (ab182858, Abcam, UK), anti-bax antibody (ab182734, Abcam), anti-CEBPB antibody (ab32358, Abcam), anti-SLC16A3 antibody (ab74109, Abcam), and anti-GAPDH antibody (ab171091, Abcam). Horseradish peroxidase-labeled IgG and enhanced chemiluminescence solution were added for visualization. With GAPDH as the loading control, immunoblots were photographed by the use of Bio-Rad image analysis system (BIO-RAD, Hercules, CA) and their densimetric analyses were performed using Quantity One v4.6.2 software.

### 2.7. Glucose Uptake, Lactate Release, and ATP Production Assays

A2780 and SKOV3 cells were seeded with 50,000 cells per well in 12-well plates and then underwent serum starvation for 24 h. Afterwards, cells were stimulated with 100 nmol/L insulin for 30 min. Cells were treated with 10 *μ*M 2-NBDG for 1 h at 37°C. The uptake of 2-NBDG was analyzed with an FC500 Flow Cytometer (Beckman Coulter, Brea, CA, USA) to reflect glucose uptake. Lactate release and ATP production were determined by Lactate Colorimetric/Fluorometric Assay Kit (BioVision, USA) and ATP Determination Kit (Thermo Fisher Scientific, USA), respectively.

### 2.8. Immunoprecipitation (RIP) Assays

A commercial kit (Millipore, USA) was used to examine the combination of LINC00035 and CEBPB following the manufacturer's manual. A2780 and SKOV3 cell lysis were centrifuged (14000 × *g*, 10 min) and cell extracts for three parts with 100 *μ*L each were collected. Immunoprecipitation was performed in two cell extracts using protein A/G sepharose beads equipped with either anti-CEBPB antibody (ab32358, Abcam) or normal mouse IgG. Immunoprecipitated RNA and total RNA from the input control were extracted for qRT-PCR analysis.

### 2.9. RNA Pull-Down Assays

A2780 and SKOV3 cells were transfected with either biotin-labeled wild-type LINC00035 or mutated LINC00035 probes for 48 h. Subsequently, cell lysis was centrifuged (14000 × *g*, 10 min). Cell extracts were immunoprecipitated with M-280 streptavidin beads (S3762, Sigma-Aldrich) precoated with RNase-free bovine serum albumin (BSA) and yeast tRNA (TRNABAK-RO, Sigma-Aldrich). Immunoprecipitated protein and total protein from the input control were extracted. Following 10% SDS-PAGE separation and membrane transfer, immunoblotting analysis of CEBPB was performed.

### 2.10. Promoter Luciferase Activity

The oligonucleotides on the 3′UTR of SLC16A3 mRNA and mutated ones were inserted into commercially available luciferase reporter vectors (pmirGLO, Promega, USA), named SLC16A3-wt and SLC16A3-mut. Treatment was done on A2780 and SKOV3 cells with SLC16A3-wt or SLC16A3-mut in the presence of CEBPB expression vector or si-CEBPB. Subsequent to 48 h of transfection, the luciferase activity in the cell lysis was determined by the dual-luciferase reporter gene assay (Promega). The relative luciferase activity was calculated using Firefly luciferase activity to ratio *Renilla* luciferase activity.

### 2.11. Chromatin Immunoprecipitation (ChIP)

To generate DNA-protein cross-links, 10% formaldehyde was added to fix A2780 and SKOV3 cells for 10 min. Chromatin fragments was generated by sonication of the DNA-protein cross-links. Three parts with equal volume were divided from the chromatin fragments. Anti-CEBPB antibody (ab32358, Abcam) or normal mouse IgG was applied to generate immunoprecipitates. Protein agarose/sepharose beads were used to precipitate the DNA-protein complexes. Cross-link and elution were finished and qRT-PCR analysis was conducted to the DNA samples. Mouse xenograft experiments.

Animal studies consisted of 12 male and 12 female BALB/c mice (Nanjing, Junke Biological Co., Ltd., Jiangsu, China), with age of 4–6 weeks and weight of 18 to 22 g. SKOV3 cells transfected with si-LINC00035 plus empty vector, si-SLC16A3, scramble siRNA plus empty vector, or si-LINC00035 plus SLC16A3 expression vector were adjusted into suspensions with 1 × 10^5^ cells/mL, and 0.5 ml of them were subcutaneously implanted into the scapular region of each mouse. The growth of xenografted tumors in mice was monitored every 5 days. When the tumor was visible by neck eyes, the length and width of the tumor were measured. After 6 weeks of implantation, the mice were euthanized by exposure to prolonged inhalational anesthesia. All animal experiments were conducted under the approval of Ethics Committee of our hospital and in accordance with the Guide for the Care and Use of Laboratory Animal. Tremendous efforts were done to minimize pain the included animals suffered from.

### 2.12. Data Analysis

SPSS 20.0 software (IBM Corp., Armonk, NY, USA) was used for statistical comparisons. A manner of mean ± standard deviation was used to display all data. Paired *t*-test was used as a statistical tool to compare data between OC tissues and nontumor tissues. One-way analysis of variance (ANOVA) was used for multiple-group comparison, and repeated measurement ANOVA was used upon different time points. A difference level less than 0.05 was indicative of statistical significance.

## 3. Results

### 3.1. LINC00035 Knockdown Attenuated Glycolysis and Apoptosis in OC Cells

The qRT-PCR demonstrated a remarkably regulated LINC00035 in OC tissues compared to that of adjacent tumor-free tissues (Figure 1(a)). Subsequently, qRT-PCR was carried out to determine the expression of LINC00035 in different OC cell lines. Similarly, we found that LINC00035 in Caov-3, A2780, SKOV3, and CoC1 human OC cell lines was increased compared with normal ovarian epithelial cells IOSE80, especially highly expressed in A2780 and SKOV3 cells (Figure 1(a)). Considering downregulated LINC00035 in OC tissues and cells, LINC00035 knockdown A2780 and SKOV3 cells, which were confirmed by the qRT-PCR (Figure 1(b)), were successfully constructed to present the function of LINC00035 in OC. Next, LINC00035 knockdown A2780 and SKOV3 cells were analyzed by CCK-8 assays, transwell assays, flow cytometric analysis, glucose uptake, lactate release, and ATP production assays. LINC00035 knockdown leading to reduced viability (Figure 1(c)), migration (Figure 1(d)), and invasion (Figure 1(e)) in A2780 and SKOV3 cells were noted. In addition, flow cytometric analysis demonstrated more apoptotic A2780 and SKOV3 cells upon LINC00035 knockdown (Figure 1(f)). Furthermore, immunoblotting analysis found declined bcl-2 expression concomitant with elevated bax expression in A2780 and SKOV3 cells with LINC00035 knockdown (Figure 1(f)). The LINC00035 knockdown A2780 and SKOV3 cells showed decreases in glucose uptake, lactate production and ATP production as compared with the scramble siRNA cells (Figure 1(g)). These results thus suggested that LINC00035 knockdown attenuated glycolysis and apoptosis in OC cells.

### 3.2. LINC00035 Increased the SLC16A3 Transcription by Recruiting CEBPB in OC Cells

Next, we retrieved the LncMAP database (http://bio-bigdata.hrbmu.edu.cn/LncMAP/) by entering LINC00035 and found LINC00035 regulates transcription factor CEBPB and its downstream gene SLC16A3 (Figure 2(a)). Then, we conducted RIP assays in A2780 and SKOV3 cells. LINC00035 enrichments were observed in that the CEBPB immunoprecipitates in A2780 and SKOV3 cells and more LINC00035 enrichments were presented after transfection with LINC00035 expression vector (Figure 2(b)). RNA pull-down followed by immunoblotting showed CEBPB could be pulled down by biotin-labeled LINC00035 probes (Figure 2(c)). Accordingly, we mapped CEBPB and SLC16A3 into the starBase database and found CEBPB and SLC16A3 were coexpressed in OC (*r* = 0.405; *p* < 0.001, Figure 2(d)). It was found elevated luciferase activity of the SLC16A3-wt in A2780 and SKOV3 cells with CEBPB overexpression and declined luciferase activity upon CEBPB knockdown (Figure 2(e)). The ChIP assays demonstrated SLC16A3 in CEBPB immunoprecipitates using anti-CEBPB rather than normal mouse IgG. Furthermore, we found more SLC16A3 was detected in CEBPB immunoprecipitates from A2780 and SKOV3 cells upon LINC00035 expression vector transfection and less detection of SLC16A3 in CEBPB immunoprecipitates upon si-LINC00035 transfection (Figure 2(f)). These results thus suggested that LINC00035 could recruit CEBPB into the SLC16A3 promoter region, thus increasing the SLC16A3 transcription.

### 3.3. The LINC00035/CEBPB/SLC16A3 Pathway Affected Glycolysis and Apoptosis in OC Cells

Next, the investigation focused on the role of SLC16A3 in OC cells. At the beginning, we mapped SLC16A3 into the GEPIA database and found SLC16A3 was highly expressed in OC tissue (Figure 3(a)). Results of qRT-PCR and immunoblotting analysis showed SLC16A3 mRNA and protein expressions were upregulated in OC tissues compared to adjacent tumor-free tissue, in four human OC cell lines compared with normal ovarian epithelial cells (Figure 3(b)). Subsequently, we performed rescue experiments by successfully delivering si-LINC00035 plus empty vector, si-SLC16A3, scramble siRNA plus empty vector, or si-LINC00035 plus SLC16A3 expression vector into A2780 and SKOV3 cells (Figure 3(c)). The qRT-PCR and immunoblotting analysis both demonstrated declined SLC16A3 mRNA and protein expressions in A2780 and SKOV3 cells following LINC00035 knockdown. As shown in Figures 4(a)–4(c), A2780 and SKOV3 cells exhibited reduced viability, migration and invasion following SLC16A3 knockdown. We also found more apoptotic A2780 and SKOV3 cells, a lower bcl-2 protein expression and a higher bax upon SLC16A3 knockdown (Figure 4(d)). It was revealed that A2780 and SKOV3 cells with SLC16A3 knockdown presented decreases in glucose uptake, lactate production, and ATP production as compared to the scramble siRNA cells (Figure 4(e)). In A2780 and SKOV3 cells concurrently treated by si-LINC00035 and SLC16A3 expression vector, we found SLC16A3 overexpression negated the effects of LINC00035 knockdown concerning no significant differences in A2780 and SKOV3 cell viability, migration, invasion, apoptosis, glucose uptake, lactate production, and ATP production between scramble siRNA plus empty vector and si-LINC00035 plus SLC16A3 expression vector. These results thus suggested that LINC00035 promoted glycolysis and cell apoptosis through CEBPB-mediated transcriptional promotion of SLC16A3.

### 3.4. The LINC00035/CEBPB/SLC16A3 Pathway Affected the Tumorigenesis of OC Cells *In Vivo*

Finally, the effect of LINC00035 on the tumorigenesis of OC cells *in vivo* was analyzed after transfected SKOV3 cells were xenografted into nude mice. The data revealed that LINC00035 knockdown and SLC16A3 knockdown were associated with inhibition of xenotransplanted tumors in nude mice (Figure 5(a)). Six weeks after implantation, the mice were euthanized by exposure to prolonged inhalational anesthesia, with tumor bodies excised. The data showed that LINC00035 knockdown and SLC16A3 knockdown could increase the weight and volume of xenotransplanted tumors in nude mice (Figures 5(b) and 5(c)). No significant difference between scramble siRNA plus empty vector and si-LINC00035 plus SLC16A3 expression vector, suggesting that SLC16A3 overexpression negated the effects of LINC00035 knockdown on the tumorigenesis of SKOV3 cells *in vivo*.

## 4. Discussion

Recent evidence indicates that high propensity of OC cells to consume and metabolize glucose by glycolysis can fuel uncontrolled growth of abnormal cells, finally leading to disease progression and chemoresistance [23]. In the case of OC, dysregulation of lncRNAs has been reported to engage in tumor growth and metastasis [24]. The obtained data revealed LINC00035 knockdown led to reduced viability migration and invasion of OC cells concurrent with an increased apoptosis, leading to decreases in glucose uptake, lactate release, and ATP production. The OC mouse model confirmed anti-tumor effect of LINC00035 knockdown on tumor growth as well. More specifically, another investigation in this study uncovered the detailed mechanism behind the action of LINC00035 in OC, namely, a regulatory network consisting of LINC00035, the transcription factor CEBPB, and downstream gene SLC16A3.

Increasing studies have begun to focus on the effects of lncRNAs, such as LINC00494, GClnc1, and SNHG17 in OC by gene regulation from aspect of transcription regulation [25–27]. Aberrant expression of LINC00035 has been reported to regulate the development and progression of various tumors, including OC, and its high expression may contribute to tumor growth and invasion. For example, Zhang et al. demonstrated LINC00035 promoter mediated by EZH2 modulates OC progression by targeting miR-133a-3p [28]. In the study of Zeng et al., they found LINC00035 governed by the EGFR pathway promotes the tumorigenesis of OC via epigenetically suppressing TIMP2 [29]. A previous study conducted by Wu and his team found LINC00035 regulation of RhoC conferred tumor-promoting effects in OC [30]. Further functional studies verified that LINC00035 knockdown could notably repress the viability, migration, and invasion of OC, induce the apoptosis, and reduce glycolysis. Accordingly, *in vivo* experiments further validated that tumor growth inhibition and tumor size reduction were related to LINC00035 knockdown. Taken together, the oncogenic functions of LINC00035 in OC was uncovered in our study.

LncRNA regulation of transcription factor to modulate the transcription of downstream genes is a novel mechanism in tumor growth and metastasis. CEBPB is one of four known members of the C/EBP family of basic region-leucine zipper transcription factors (CEBPA, CEBPB, CEBPD, and CEBPE) [31]. The transcriptional regulation of CEBPB on downstream genes is regulated by lncRNA in human diseases. For example, Wu et al. demonstrated LINC00160 mediated acquired resistance of chemotherapeutic regimes of paclitaxel and doxorubicin drugs in breast cancer cells by regulating TFF3 via transcription factor C/EBP*β* [32]. Gao et al. found that silencing of lncRNA LEF1-AS1 reduced EZH2 expression to repress hepatocellular carcinoma progression by disruption of CEBPB interaction with CDCA7 [33]. Only a previous study investigates the role of CEBPB in the case of OC that CEBPB expression was not significantly changed in OC tissues and cells, which was partially consistent with our results that CEBPB was just responsible for the regulation of LINC00035 on the SLC16A3 expression in OC.

SLC16A3 is greatly involved in tumor pH modulation as a lactate transporter. In a mouse tumor model, lactate modulation and anti-tumor activity were evaluated through the direct target interaction of the optimized compound 18n with the cytosolic domain of SLC16A3 suggesting pharmacokinetic inhibition of SLC16A3 by 18n is a useful outcome measure for anti-tumor effects on tumor biology [34]. Our following investigations demonstrated SLC16A3 was upregulated in OC tissues. SLC16A3 knockdown exerted similar effects on SKOV3 and A2780 cells as LINC00035 knockdown, especially attenuating glucose uptake, lactate production, and ATP production. In a gliomas report, Reuss et al. indicated that the function SLC16A3 is lactate and proton exporter. The expression of SLC16A3 was negatively correlated with extracellular pH and proportional to extracellular lactate concentrations [35]. Yu and his team performed integrated bioinformatics that comprehensively analyzed the SLC16A gene family in pancreatic cancer, showing SLC16A exhibited biomarker potential for prognosis of pancreatic cancer [36]. Concurring with our data concerning SLC16A3 expression in OC, SLC16A3 was remarkably increased in liver cancer [37].

In summary, the study mainly highlights a new mechanism by regulating the transcription factor CEBPB and the downstream genes SLC16A3 to confirm the function of LINC00035 in OC. LINC00035 acts as an oncogenic lncRNA in OC tumorigenesis. The finding revealed in this study may confer valuable view to develop new therapeutic targets for OC (Figure 6). The interaction between LINC00035, CEBPB, and SLC16A3 needs to be further studied to deeply understand and clarify the specific mechanisms related to antiglycolysis action of SLC16A3 in OC, in order to verify its application value from the perspective of clinical practice.

## Figures and Tables

**Figure 1:** LINC00035 knockdown attenuates glycolysis and apoptosis in OC cells. (a) Expression of LINC00035 in OC tissues (*n* = 67), adjacent tumor-free tissues (*n* = 67), ovarian epithelial cells, and OC cell lines determined by RT-qPCR. (b) Validation of LINC00035 knockdown A2780 and SKOV3 cells. (c) Reduced A2780 and SKOV3 cells following LINC00035 knockdown. (d, e) Fewer A2780 and SKOV3 cells transferring from the apical chamber of the transwell system uncoated or coated with Matrigel into the basolateral chamber following LINC00035 knockdown. (f) Immunoblots and quantification of bcl-2 and bax in A2780 and SKOV3 cells following LINC00035 knockdown. (g) Decreases in glucose uptake, lactate production, and ATP production in A2780 and SKOV3 cells following LINC00035 knockdown. ^*∗*^*p* < 0.05.

**Figure 2:** LINC00035 increases the SLC16A3 transcription by recruiting CEBPB in OC cells. (a) LINC00035 regulation of SLC16A3 via transcription factor CEBPB is predicted in the LncMAP database. (b) RIP-qPCR examined the LINC00035 in CEBPB immunoprecipitates from A2780 and SKOV3 cells with or without LINC00035 overexpression. (c) RNA pull-down followed by immunoblotting analysis examined the CEBPB pulled down by biotin-labeled LINC00035 probes. (d) Coexpression between CEBPB and SLC16A3 in the starBase database. (e) Dual-luciferase reporter gene assays to validate SLC16A3 binding with CEBPB in A2780 and SKOV3 cells. (f) ChIP assays followed by immunoblotting analysis examined the SLC16A3 in CEBPB immunoprecipitates from A2780 and SKOV3 cells with or without LINC00035 knockdown ^*∗*^*p* < 0.05.

**Figure 3:** LINC00035 increases SLC16A3 expression in OC cells. (a) SLC16A3 was highly expressed in OC tissue in the GEPIA database. (b) SLC16A3 expressions in OC tissues and cells, measured by qRT-PCR and immunoblotting analysis. (c) si-LINC00035 plus empty vector, si-SLC16A3, scramble siRNA plus empty vector, or si-LINC00035 plus SLC16A3 expression vector were delivered into A2780 and SKOV3 cells and qRT-PCR, and immunoblotting analysis were used to determine SLC16A3 mRNA and protein expressions ^*∗*^*p* < 0.05.

**Figure 4:** The LINC00035/CEBPB/SLC16A3 pathway affects glycolysis and apoptosis in OC cells. (a) CCK-8 assays examined A2780 and SKOV3 cells upon SLC16A3 knockdown or LINC00035 knockdown and SLC16A3 overexpression concurrently. (b, c) Representative view and statistics of A2780 and SKOV3 cells transferring from the apical chamber of the transwell system uncoated or coated with Matrigel into the basolateral chamber upon SLC16A3 knockdown or LINC00035 knockdown and SLC16A3 overexpression concurrently. (d) Immunoblots and quantification of bcl-2 and bax in A2780 and SKOV3 cells upon SLC16A3 knockdown or LINC00035 knockdown and SLC16A3 overexpression concurrently. (e) Glucose uptake, lactate production, and ATP production measurements in A2780 and SKOV3 cells upon SLC16A3 knockdown or LINC00035 knockdown and SLC16A3 overexpression concurrently ^*∗*^*p* < 0.05.

**Figure 5:** The LINC00035/CEBPB/SLC16A3 pathway affects the tumorigenesis of OC cells in vivo. (a) Subcutaneously xenografted tumors. (b) Tumor weight. (c) Tumor growth ^*∗*^*p* < 0.05.

**Figure 6:** A schematic diagram showing how the LINC00035/CEBPB/SLC16A3 pathway regulates the development of OC. LINC00035 was triggered in OC and could recruit the transcription factor CEBPB into the SLC16A3 promoter region, thus increasing the SLC16A3 transcription. Abundance of SLC16A3 inhibited OC cell viability, migration, invasion, and glycolysis and induced the apoptosis.

## Data Availability

The data used for this study were included in the article.
